The article "The role of ICT investment, digital financial inclusion, and environmental tax in promoting sustainable energy development in the MENA region: Evidences with Dynamic Common Correlated Effects (DCE) and instrumental variable-adjusted DCE" was retracted in 2025. Reasons: unreliable results or conclusions; citations of retracted work; concerns about the article.

# The role of ICT investment, digital financial inclusion, and environmental tax in promoting sustainable energy development in the MENA region: Evidences with Dynamic Common Correlated Effects (DCE) and instrumental variable-adjusted DCE

**DOI:** 10.1371/journal.pone.0301838

**Published:** 2024-05-06

**Authors:** LIU Xiangling, Md. Qamruzzaman

**Affiliations:** 1 School of Business, Hunan University of Science and Technology, Hunan, China; 2 School of Business and Economics, United International University, Dhaka, Bangladesh; The University of Dodoma, UNITED REPUBLIC OF TANZANIA

## Abstract

His research investigates the interplay among investment in Information and Communication Technology [ICT], digital financial inclusion, environmental tax policies, and their impact on the progression of sustainable energy development within the Middle East and North Africa [MENA] region. Recognizing the distinctive hurdles impeding sustainable energy advancement, effective policy formulation and implementation in MENA necessitate a comprehensive understanding of these variables. Employing a Dynamic Common Correlated Effects [DCE] model alongside an instrumental variable-adjusted DCE approach, this study explores the relationship between ICT investment, digital financial inclusion, environmental tax, and sustainable energy development. The DCE model facilitates the analysis of dynamic effects and potential correlations, while the instrumental variable-adjusted DCE model addresses issues pertaining to endogeneity. The results indicate that both ICT investment and the promotion of digital financial inclusion significantly and positively impact sustainable energy development in the MENA region. Additionally, the study underscores the importance of environmental tax implementation in fostering sustainable energy advancement, highlighting the critical role of environmental policy interventions. Based on these findings, governmental prioritization of ICT investment and initiatives for digital financial service integration is recommended to bolster sustainable energy growth in MENA. Furthermore, the adoption of efficient environmental tax measures is essential to incentivize sustainable energy practices and mitigate environmental degradation. These policy recommendations aim to create a conducive environment for sustainable energy progression in the MENA region, contributing to both economic prosperity and environmental conservation.

## I. Introduction

Clean energy is essential for alleviating environmental issues, providing a sustainable substitute for fossil fuels, and diminishing greenhouse gas emissions globally Mac Kinnon, Brouwer [1]. The necessity to embrace renewable energy is founded upon its capacity to mitigate climate change, bolster energy security, and stimulate economic expansion. Nevertheless, the achievement of this potential is impeded by various challenges, such as restricted financial resources available for renewable energy initiatives, specifically in underserved communities Ali, Jianguo [2]. With the decreasing cost of renewable energy technology, it is becoming increasingly competitive compared to conventional fossil fuels. This cost reduction leads to lower energy expenses for businesses and individuals, freeing up financial resources for other investments and promoting economic growth [3–9]. The renewable energy sector is a rapidly growing industry with great promise for job creation and economic growth. Based on the International Energy Agency [IEA] findings, the renewable energy sector is estimated to create an additional 28 million job opportunities globally by 2050. The nations in the MENA region, known for their significant and growing young populations, have the potential to capitalize on this opportunity to enhance job creation and address the issue of unemployment. Furthermore, adopting clean energy can potentially support nations in the Middle East and North Africa [MENA] region in diversifying their economic activities, reducing their dependence on oil and gas exports and enhancing their resilience to fluctuations in global energy prices.

The Middle East and North Africa [MENA, hereafter] area is noted for its high per capita energy consumption, which exceeds the world average and may be attributable to various things. One is the region’s hot and dry environment, which necessitates air conditioning. Furthermore, the availability of oil and gas resources in the region has resulted in a long-term dependence on fossil fuels as the major energy source. There has been a growing trend toward renewable energy usage in the MENA area in recent years. Several reasons contribute to this tendency, including increasing costs connected with fossil fuels, growing awareness about climate change, and a desire to reduce dependence on foreign energy supplies. The MENA area is now seeing a considerable surge in the use of renewable energy sources for various reasons. The region’s installed renewable energy capacity increased significantly in 2022, reaching 28.5 gigatonnes [GW]. This marks a significant 25% gain over the previous year. Iran has the area’s most installed renewable energy capacity, at over 12 GW. The UAE and Saudi Arabia are closely following suit in this admirable initiative. Renewable energy is expected to increase steadily in the MENA area shortly. According to the International Energy Agency [IEA], the region’s renewable energy capacity is expected to reach 100 GW by 2030. Several main variables will contribute to the predicted rise in the renewable energy industry in developing nations including [10–15]. The government’s adoption of policies promoting the growth of renewable energy sources is among the most crucial components. Located at a critical juncture in energy, the MENA area is confronted with a clear-cut decision: either completely abandon fossil fuels, which contribute substantially to air pollution and global warming or diversify its energy portfolio.

Additionally, it might choose renewable energy, improving its inhabitants’ future. Immediately transitioning to renewable energy sources is essential for the Middle East and North Africa [MENA] region to safeguard its population and the environment for future generations. Numerous factors influence the pace of adoption of renewable energy. The energy market is subject to the effect of many elements, including but not limited to technical improvements, financial incentives, public mood and comprehension, energy pricing, the availability of renewable energy infrastructure, and market dynamics [16–18]. Various governmental rules and regulations, such as carbon pricing, renewable energy targets, and tax incentives for producing and using clean energy, substantially influence the transition towards renewable energy sources. Proximity technology improvements may facilitate the imminent enhancement of the accessibility and cost-effectiveness of renewable energy sources such as solar, wind, and hydropower. Consequently, this may lead to an increase in their use. Environmentally friendly energy project-specific subsidies and tax credits are economic incentives that might be implemented to promote the use of renewable energy sources.

The present study has considered investment in ICT, digital financial inclusion [DF, hereafter], and environmental tax [ET, hereafter] in the equation of clean energy consumption in MENA countries for 2004–2019. Amid this complex environment, the study of digital finance arises as a strategic pathway. By its pioneering technologies and all-encompassing frameworks, digital finance has the potential to fundamentally transform the financial sector and enhance the availability of capital for renewable energy endeavours solutions Kor and Qamruzzaman [19]. Digitalization has also safeguarded the animals using distinctive and advanced tactics Raiaan, Fahad [20]. Through an analysis of the combination of renewable energy and digital finance, this study aims to understand the intricate correlation between the environmental sustainability implications of digital platform-enabled financial inclusion and digital finance Macchiavello and Siri [21]. Comprehending this correlation is crucial for evaluating the potential of digital financial inclusion to close financial disparities, encourage investments in renewable energy, and foster a more environmentally aware global economy Wang, Sun [22]. This study aims to identify potential advantages and obstacles while examining this intricate relationship. The findings will ultimately contribute to developing policies and approaches that utilize digital finance to hasten the worldwide shift towards environmentally friendly and sustainable energy sources. By delving into the connection between digital finance and clean energy, we can tackle the issue of financial accessibility gaps while harnessing technology’s transformative power Salampasis and Mention [23]. By incorporating digital tools into clean energy initiatives, we aim to make financial access more accessible, enhance efficiency, and encourage the widespread adoption of sustainable energy. This will contribute to achieving global sustainability objectives in an ever-evolving digital landscape [24–27].

The study is motivated by the existing literature and intended to fill the gap with empirical findings. First, the effects of ICT and digital finance are immensely important for economic and environmental sustainability, as documented in the literature. On the other hand, in the case of energy transition, the roll of DF has yet to be extensively assessed and properly documented, especially in the case of MENA nations; it is still uncovered in the empirical investigation. Thus, the present study has initiated an exploration of fresh evidence through empirical investigation and offers fresh evidence in the existing literature. The findings suggest that digital financial technologies, such as block chain, mobile payment systems, and big data analytics, play a vital role in expanding the accessibility of green finance options for renewable energy projects. The report highlights the importance of continued government support in developing digital financial infrastructure to foster a sustainable and eco-friendly energy framework. Digital finance plays a crucial role in promoting financial transparency, facilitating the creation of innovative financial instruments like green bonds and carbon credits, and broadening the availability of funds for clean energy projects. This, in turn, accelerates the advancement and implementation of renewable energy initiatives. Extensive research supports the idea that when economic incentives are aligned with environmental goals, it can effectively steer the energy market towards cleaner alternatives.

This research is driven by the pressing need to address the challenges of sustainable energy development in the MENA region. Considering the increasing global concern regarding climate change and the depletion of traditional energy sources, countries in the MENA region must transition towards sustainable energy alternatives. This research aims to examine the potential impact of investments in ICT [Information and Communication Technology], digital financial inclusion, and environmental tax on the progress of sustainable energy development in the MENA region. By understanding the importance of these factors, policymakers and stakeholders can make informed decisions to advance sustainable energy projects and contribute to global environmental sustainability. The study’s significance lies in its capacity to offer valuable insights into the complex interplay among ICT investment, digital financial inclusion, environmental tax laws, and sustainable energy growth in the MENA region. The research seeks to gain a comprehensive understanding of the opportunities and limitations associated with the transition to sustainable energy sources through a detailed analysis of these factors. The findings of this study could offer significant insights for the development of targeted regulations, investment strategies, and technological advancements aimed at accelerating the adoption of sustainable energy solutions in the MENA region. Ultimately, the significance of this study lies in its potential to contribute to the global effort of mitigating climate change and promoting sustainable development in the MENA region and beyond. The contribution of the study is as follows;

First, Studies have indicated that digital finance has the potential to expand the accessibility of eco-friendly financing options for renewable energy projects, especially in developing countries [28]. Digital finance facilitates transparent financing options, promotes innovative financial technologies’ advancement, and enhances funds’ availability for sustainable energy projects [29, 30]. Digital financial technology enables transparent and secure transactions, while mobile payment solutions improve financial service accessibility in rural regions. In addition, using big data analytics can assist in identifying investment opportunities and assessing the environmental impact of projects [16, 31]. This study explores the potential benefits and challenges of adopting digital financial inclusion and their impact on promoting sustainable energy.

The second contribution deals with the research that emphasizes the critical significance of Information and Communication Technology [ICT] in enabling the seamless incorporation of renewable energy sources into the existing energy framework. As the literature gap suggests, consumers can make environmentally conscious and well-informed energy decisions by implementing efficient communication systems and cutting-edge technologies. ICT-enabled smart metering systems allow consumers to monitor their energy usage, identify possible areas for enhancement, and make informed choices regarding adopting renewable energy sources [32–35]. Furthermore, ICT solutions can automate energy-conservation strategies, efficiently coordinating energy usage with the accessibility of renewable energy. Ultimately, this enhances the prospect of a more sustainable future. The research emphasizes ICT’s critical role in developing consumer engagement platforms that motivate and educate individuals regarding adopting renewable energy usage. This encompasses the progression of virtual power plants capable of integrating a diverse range of renewable energy sources [19, 27, 36–40].

Third, Based on the findings, it is evident that environmental levies play a significant role in promoting the adoption of renewable energy sources. By implementing taxation on activities that harm the environment, governments can foster the adoption of cleaner practices and stimulate the advancement and utilization of renewable energy sources [31]. Tax credits and incentives are critical for promoting the broad use of renewable energy sources and attracting significant investments in environmentally beneficial projects [30]. Extensive research supports the premise that combining economic incentives with environmental goals might help steer greener energy sources more successfully. Several studies have shown that environmental levies are important in encouraging the adoption of renewable energy sources in industrialized and rich countries. On the other hand, their effects on emerging nations are more complicated and harder to predict. Numerous studies, backed up by environmental fees, predict a huge increase in the usage of renewable energy sources in wealthy countries [29]. However, it must be understood that different taxes may affect developing nations differently, resulting in different results. Environmental taxes, to a considerable degree, aid in preventing environmental damage by giving cash for investments in renewable energy and ecologically responsible governance [41]. Furthermore, environmental levies are particularly successful in reducing greenhouse gas emissions and supporting the expansion of renewable energy sources. Overall, this research illustrates the possible advantages and downsides of environmental taxation and its capacity to stimulate the use of renewable energy sources [42, 43].

The rest of the structure is as follows. Section II deals with the survey of pertinent literature, the data and methodology of the study exhibited in Section III, empirical model estimation and interpretation reported in Section IV, Section V deals with the discussion of the study findings and the conclusion and policy suggestions available in Section VI, respectively.

## II. Literature reviewer

### 2.1 ICT and clean energy nexus

Studies have shown much interest in looking at how ICT affects the use of renewable energy sources. How digital currency could affect renewable energy consumption and energy efficiency has been the subject of a great deal of study [44–50]. Based on a study conducted by researchers [51], it has been found that the utilization of Information and Communication Technology [ICT] in conjunction with renewable energy sources has the potential to effectively diminish and replace the reliance on traditional fossil fuels. However, it is important to note that ICTs consume significant energy, particularly during the operation or installation of equipment that relies on electricity. As a result, this can lead to an increase in overall energy demand [52]. According to the study, using ICT-related applications, including social media, laptops, and smartphones, has resulted in a rise in energy consumption associated with ICT in the residential sector. The objective of a subsequent study [53] was to ascertain whether using ICT in conjunction with renewable energy sources has the potential to enhance environmental quality. According to the study, the integration of ICT and renewable energy has the potential to contribute significantly to sustainable development. This can be achieved through the reduction of greenhouse gas emissions, the promotion of energy efficiency, and the enhancement of resource utilization. According to the report, in 2014, a total of 17% of the electricity consumption within the ICT industry was sourced from renewable sources. Moreover, the utilization of information and communication technology [ICT] in the process of transitioning to renewable energy sources is also emphasized in a report4. The report posits that the utilization of IoT-enabled devices holds the potential to mitigate energy consumption within smart networks, primarily through the implementation of logistics applications. According to a report from the U.S. Department of Energy, implementing interactive ICT across all power generation sources can effectively optimize the utilization of the most cost-effective or renewable energy in real-time [35].

The of significant potential for ICT in the energy sector and their role in achieving Sustainable Development Goal 7; additionally, ICT can promote energy conservation and efficiency by implementing sensing and control mechanisms [44, 45, 47, 50, 54, 55]. ICT has the potential to enhance resource utilization through the implementation of shared systems and the promotion of efficiency, facilitated by intelligent appliances, infrastructure, and production methods. In the study [56, 57], the ICT sector has the potential to drive the renewable energy revolution by achieving a 20% reduction in emissions by 2030. This can be accomplished through the intelligent application of ICT in improving energy efficiency in the transportation, energy, and real estate sectors. Integrating information and communication technology [ICT] with renewable energy holds significant potential in fostering sustainable development. This potential lies in its ability to effectively reduce greenhouse gas emissions, promote energy efficiency and enhance resource utilization. Nevertheless, using ICT also requires energy, potentially escalating the overall demand. The ICT sector is a noteworthy consumer of renewable energy as well. Moreover, the utilization of IoT-enabled devices holds the potential to effectively curtail energy consumption within smart networks [50, 55].

### 2.2 Digital financial inclusion and clean energy

The study of [58] examined the impact of digital finance on energy efficiency in China. It has been discovered that digital finance has the potential to have a significant impact on energy efficiency. This is primarily due to its critical role in resource allocation and risk management. However, the study also identified potential challenges that may arise from network externalities, which could result in the monopolization of the digital finance industry. This monopoly has the potential to impede energy efficiency enhancements through the generation of resource mismatches, suppression of innovation, and facilitation of corrupt practices. Therefore, it is crucial to comprehend the intricate relationship between digital finance and energy efficiency, especially within the framework of attaining global sustainable development goals. A similar study can be found in the study of [59]. The study unveiled a favourable influence of digital finance in facilitating the uptake of renewable energy consumption. The study emphasizes that implementing digital finance plays a crucial role in promoting the development above by effectively addressing information asymmetry, minimizing transaction costs, and alleviating financing constraints within the renewable energy sector. Therefore, the emergence of digital finance is a promising catalyst for advancing renewable energy deployment, significantly contributing to establishing a more sustainable energy landscape. In this report, [60] analyzes the intersection of digital finance and energy efficiency to provide a comprehensive overview of the current state of digital finance regarding energy efficiency and identify potential opportunities and challenges in this field. The study identified multiple mechanisms by which digital finance can effectively reduce energy consumption. These encompass the optimization of resource allocation, the promotion of technological innovation, the facilitation of knowledge spillovers, and the provision of platforms for energy-saving services. The report highlights the potential of digital finance to enhance energy efficiency and address climate change, aligning with sustainable development objectives.

The study of [61] analyzes digital finance’s collective impact on renewable energy consumption and CO2 emissions. The study’s findings indicate a positive correlation between the heightened utilization of digital finance, elevated levels of renewable energy consumption, and decreased CO2 emissions. The findings underscore the potential of digital finance as a pivotal catalyst for sustainable development. This is evident in its ability to not only promote the adoption of renewable energy but also to aid in the reduction of greenhouse gas emissions. This is primarily achieved through the promotion of renewable energy adoption, the enhancement of energy efficiency, and the reduction of greenhouse gas emissions. However, the magnitude of this impact is contingent upon many factors, encompassing network externalities, financing constraints, and regional disparities. A comprehensive comprehension of these intricacies can facilitate the development of efficient policies and strategies aimed at maximizing the potential of digital finance in promoting the sustainable advancement of clean energy in China and other regions.

Zhou, Zhang [62] stated a decline in household carbon emissions has been observed due to digital financial inclusion, specifically in urban regions, via electricity consumption and the proportion of renewable energy usage. Ali, Jianguo [2] discovered that the correlation between environmental sustainability and economic growth has been established, with digital financial inclusion concurrently fostering sustainable social and economic development by expediting the adoption of renewable energy sources and promoting energy diversification. Likewise, inclusive digital finance effectively mitigates carbon emissions by providing diversified financial products to investors, thereby substantially augmenting the funding available for renewable energy initiatives, as claimed by Liu, Yao [63]. Macchiavello and Siri [21] also ascertained digital finance has the potential to facilitate investments in environmentally conscious enterprises and initiatives, thus promoting sustainable practices and aiding in the expansion of the green economy. Raiaan, Fatema [64] also found that digital financial inclusion leads to advanced healthcare opportunities. Consequently, people become more aware and conscious about themselves and externalities. Moreover, Yu, Wei [65] also demonstrated that advocating for digitally accessible green finance contributes to developing green and renewable energy resources and reducing CO2 emissions. Additionally, Han, Li [66] discovered that the optimization of green development efficacy is facilitated by digital finance, and the interaction between digital finance and environmental regulation yields favourable results for green development. Digital financial inclusion promotes green economic efficiency through the following mechanisms: reduction of information asymmetry, facilitation of loan acquisition for small innovative enterprises engaged in green innovation, and augmentation of investment in environmentally sustainable modes of consumption, unveiled by [67]. Salman and Ismael [68] revealed that promoting online digital payment gateways and increasing consumer awareness regarding the significance of going green are two ways digital financial inclusion encourages consumer participation in environmental protection activities. This can result in a reduction in paper-based transactions and facilitate the transition to cashless societies. França, Neto [69] revealed that adopting digital financial services results in a diminished reliance on paper-based transactions, promoting environmental conservation and reducing paper usage. Similarly, Berkhout and Hertin [70] also unearthed digital finance inclusion significantly reduces transaction costs and eliminates many environmental costs associated with paper-based transactions and ICTs contribute significantly to structural changes.

The subsequent evidence highlights the adverse linkage between digital finance/ digital financial inclusion and environment and clean energy. In some instances, Galanti and Ӧzsoy [71] said that digital financial inclusion has increased carbon dioxide emissions, particularly in developing nations, where the rapid expansion of the digital finance sector contributes to climate change. Zheng and Li [72] proclaimed as more individuals and organizations depend on digital platforms for transactions and other services, using digital financial services may result in heightened energy consumption. This may counterbalance the potential environmental benefits of digital finance, such as reducing carbon emissions. Sun, Hu [73] said the proliferation of digital finance may result in resource depletion due to the augmented energy and raw material demands that support digital infrastructure and services. This, in turn, may contribute to environmental degradation. Tansel [74] found that expanding digital finance may give rise to heightened waste generation due to the production and disposal of electronic devices and infrastructure, which subsequently contribute to environmental degradation. Likewise, Premalatha, Tabassum-Abbasi [75] found that it is recycled or dumped without concern that gross pollution is caused. The problem is increasing much faster than the efficacy of our strategies to contain it. La Torre, Dumay [76] claimed that the digital financial industry is susceptible to security threats and data privacy violations, potentially compromising personally identifiable information and impeding environmental initiatives to safeguard sensitive data. An older study by Azmi, Zulhuda [77] documented that the world is becoming more vulnerable to data breaches. Its compromise can have far-reaching consequences and undermine public safety and social and environmental threats. Awasthi and Li [78] also revealed that environmental pollution can result from producing and disposal of electronic devices and infrastructure, which may increase electronic refuse as digital finance expands. Also, as an increasing number of individuals and organizations depend on digital platforms for conducting transactions and accessing additional services, implementing digital financial services may result in heightened energy consumption. This could counterbalance the advantages of digital finance regarding carbon emission reduction, stated by Ren, Hao [79]. Sharma and Dash [80] found that the expansion of digital finance may result in a corresponding rise in carbon footprint due to the energy consumption necessary to operate digital infrastructure and devices.

### 2.3 Theoretical and conceptual framework of the study

To achieve sustainable growth, it is crucial to comprehend the intricate interaction of several components. The objective of this research is to examine the connections between investment in information and communication technology [ICT], digital financial inclusion [DFI], and environmental taxes and their collective influence on the advancement of sustainable energy development [SED]. The theoretical and conceptual framework serves as the basis for this study, providing a clear guide for understanding the complex dynamics involved.

The Sustainable Development Theory, which emphasizes the interdependence of economic, social, and environmental aspects in achieving sustainability, serves as the research’s guiding principle. This theory guides the investigation of the combined impact of ICT, DFI, and environmental taxes on sustainable energy development. In addition, the research utilizes the theoretical framework of technological determination to analyze the influential impact of ICT investment on altering the energy landscape. From this standpoint, technology is a potent influence that moulds social frameworks and actions. Within the framework of this research, investment in information and communication technology [ICT] is seen as a stimulant for promoting innovation and effectiveness in the energy industry [52]. This, in turn, encourages the adoption of sustainable practices and the use of renewable energy sources. The concept of digital financial inclusion is examined from the perspective of financial inclusion theory, which highlights the significance of giving consumers and companies cheap and efficient access to financial services [81]. Digital Financial Inclusion [DFI], enabled by digital technology, is anticipated to improve financial accessibility, particularly in the realm of sustainable energy initiatives [82–84]. This theory facilitates the analysis of how DFI might enable communities to engage in and get advantages from sustainable energy efforts [2]. The research further integrates environmental taxation theory to examine the impact of policy tools on fostering sustainable activities. Environmental taxes are seen as tools for internalizing external costs and promoting environmentally conscious actions. This theory facilitates comprehension of how the implementation of environmental levies might impact enterprises and consumers, prompting them to make decisions that are in line with sustainable energy development objectives.

Within the conceptual framework, ICT investment is positioned as a pivotal factor that significantly impacts sustainable energy development. The integration of technology into the energy industry is anticipated to bolster grid management, optimize energy efficiency, and streamline the incorporation of renewable energy sources. DFI plays a crucial role in advancing sustainable energy development by ensuring that financial services are available to all stakeholders, particularly those in distant and disadvantaged regions. Digital platforms provide consumers and organizations with access to financial instruments that may assist their participation in sustainable energy initiatives. The Environmental Tax is included in the framework as a regulatory tool that promotes environmentally conscious behaviour. The core of the conceptual framework is sustainable energy development, which represents the ultimate objective of the research. Sustainable Energy Development [SED] involves the use of renewable energy sources, enhanced energy efficiency, and the overall mitigation of environmental harm. The integration of ICT Investment, DFI, and Environmental Tax is anticipated to merge on SED, generating a synergistic impact that drives the energy industry towards a sustainable future.

## III. Material and methods

### 3.1 Empirical model construction and specification

The motivation of the study is to gauge the impact of investments in ICT, digital financial inclusion, and environmental tax on clean energy in the MENA region, consisting of a panel of 17 nations for the period 2004–2019. The empirical model exhibits the relations between explained and explanatory variables and three control variables.


Model1:CE∫ICT,GF,ET [1]

Model2:CE∫ICT,GF,ET,FO,TO,EQ [2]

With log transformation, the above Eq [1] and Eq [2] can be reproduced in a regression form in the following manner.


$$Model-01:\;{CE}_{it}=\beta_{0}+\beta_{1}{ICT}_{it}+\beta_{2}{GF}_{it}+\beta_{3}{ET}_{it}+\epsilon$$ [3]

$$Model\;02:\;{CE}_{it}=\beta_{0}+\beta_{1}{ICT}_{it}+\beta_{2}{GF}_{it}+\beta_{3}{ET}_{it}+\beta_{4}{FO}_{it}+\beta_{5}{TO}_{it}+\beta_{6}{EQ}_{it}+\epsilon$$ [4]

For ICT investment, it is anticipated that the coefficient of β_1_>0, that is, the ICT coefficient demonstrates a positive link between the degree of infrastructure and usage of information and communication technology [ICT] and the adoption of renewable energy technologies, which means that a greater degree of ICT may help to improve the adoption of renewable energy solutions, due to improved information availability, more effective communication channels for exchanging experiences and best practices, and the emergence of novel clean energy solutions [85, 86]. According to the coefficient on digital financial inclusion, it is expected to be positive and statistically significant. That is the availability and use of digital financial systems, such as mobile payment systems and cryptocurrencies, might stimulate the uptake of clean energy solutions. This might be because these technologies make it simpler to get finance and lessen the financial barriers associated with embracing sustainable energy. The coefficient of β_3_>0, implying that environmental taxes increasing taxes on activities that affect the environment may serve as an incentive for the adoption of greener energy technology. This is due to the idea of internalizing environmental externalities, which entails people and corporations accepting full responsibility for the costs connected with their activities. This method supports the adoption of more environmentally friendly options.

### 3.2 Variables definition and anticipated sign of coefficients

The term "information and communications technology" [ICT] refers to the essential structure and components that make contemporary computing possible. The term "information technology" [IT] refers to a wide range of components, including applications, communication devices, and networking components respectively. A number of capabilities, including the coordination, administration, protection, transmission, and exchange of data and information, are made possible by it [1, 2, 4]. ICT stands for "information and communication technologies," which encompasses a wide variety of technological instruments and resources that are used for the purpose of transmitting, storing, generating, sharing, or exchanging data. The telephone, computers, the Internet, live and recorded broadcasting technologies, and telephony are all examples of technology that fall under this category. The goals of information and communications technology [ICT], which are always evolving, include enhancing the ways in which people generate, process, and exchange data or information, as well as enhancing abilities in a wide variety of fields, including business, education, medicine, and the ability to solve practical problems. The term "digital world" refers to the collection of gadgets, networking components, and applications that all work together to make it possible for individuals and organizations to communicate with one another.

Digital Financial Inclusion [DFI] has the potential to positively impact the use of sustainable energy via many means. Firstly, it can reduce the expenses associated with conventional banking, therefore simplifying the procedure of obtaining financial services and making them more cost-effective for people and businesses. Over time, this might result in a decrease in pollution levels by promoting investment in eco-friendly infrastructure and renewable energy sources. Furthermore, DFI can enhance the availability of clean energy initiatives, therefore facilitating a larger proportion of households to get financial support for their involvement in clean energy endeavours. As a result, this could lead to the substitution of devices currently utilizing energy, the enhancement of the energy consumption balance, and a rise in the utilization of renewable and recycled energy sources, ultimately resulting in improved energy efficiency. Moreover, DFI can enhance public awareness about the environment and stimulate societal investment in renewable energy sources. Consequently, this aids in mitigating environmental impacts and promoting the achievement of sustainable development goals. Furthermore, the implementation of inclusive digital finance can provide investors with a diverse array of financial options, therefore significantly augmenting the available funds for environmentally sustainable technology initiatives and mitigating carbon dioxide emissions. The last aspect to consider is that the impact of digital financial inclusion [DFI] on the adoption of renewable energy might vary across different regions and between urban and rural areas. Policymakers may use this information to develop regionally suitable and effective strategies to advance digital financial inclusion and boost the adoption of renewable energy. The realm of digital finance possesses the inherent capacity to enhance the scope of financial inclusion, facilitate enhanced accessibility to financial services, and elevate the overall efficiency of the financial sector. The proxy variables of DFI are posted in Table 1.

**Table 1:** Proxy variables of digital financial inclusion.

Notation	Proxy	Data sources
DF1	Number of ATMs per 1.000 km2	International Financial Statistics—IMF
DF2	Number of ATMs per 100.000 adults	
DF3	Number of Deposit Accounts with	
DF4	Commercial Banks per 1000 adults	
DF5	Number of commercial bank branches per 1.000 km2	
DF6	Number of commercial bank branches per 100.000 adults	
DF7	Outstanding deposits with commercial banks [% of GDP]	
DF8	Outstanding loans from commercial banks [% of GDP]	
Df9	Account ownership at a financial institution or with a mobile-money service provider [% of the population ages 15+]	World development indicator

The study has implemented the PCA in constructing the index of digital financial inclusion [DFI], and the detailed results of factors contributing to the index are displayed in Table 2

**Table 2:** Results of principal components analysis.

Number	Value	Difference	Proportion	CV	CP				
1	3.3113	2.0821	0.3679	3.3113	0.36799				
2	1.2292	0.26058	0.1365	4.5406	0.5045				
3	0.9686	0.0832	0.1076	5.5092	0.6121				
4	0.8853	0.2645	0.0983	6.3946	0.7105				
5	0.6208	0.0151	0.0689	7.0154	0.7794				
6	0.6056	0.0817	0.0672	7.6211	0.8467				
7	0.5238	0.0325	0.0582	8.14502	0.9050				
8	0.4913	0.1277	0.0545	8.6364	0.9598				
9	0.3635	---	0.0403	9	1				
Eigenvectors [loadings]:									
Variable	PC 1	PC 2	PC 3	PC 4	PC 5	PC 6	PC 7	PC 8	PC 9
1	0.2603	0.5663	-0.0124	0.4973	0.3083	-0.11345	0.1099	0.0516	0.4912
2	0.3263	0.4837	0.3267	0.0671	-0.2030	0.2281	-0.4298	0.0401	-0.5182
3	0.3189	-0.3285	-0.0374	0.4956	-0.2524	0.5264	0.4219	-0.1241	-0.0942
4	0.3728	0.1569	-0.0464	-0.5183	-0.1619	0.1640	0.0353	-0.6275	0.3425
5	0.3459	-0.3105	-0.4133	-0.0207	0.1921	0.2721	-0.6031	0.2898	0.2319
6	0.2985	-0.1565	0.6005	-0.3534	0.3325	0.1556	0.2753	0.4199	0.1169
7	0.3298	-0.3908	0.2467	0.2388	0.3414	-0.4795	-0.1854	-0.4483	-0.1962
8	0.3850	-0.0932	-0.0095	-0.0107	-0.6527	-0.5283	0.0495	0.3330	0.1557
9	0.3451	0.1739	-0.5449	-0.2265	0.2892	-0.1535	0.3838	0.1189	-0.4833
1	1								
2	0.47284	1							
3	0.18472	0.1917	1						
4	0.20806	0.4088	0.2167	1					
5	0.1101	0.1683	0.3944	0.3314	1				
6	0.0857	0.3023	0.2304	0.3457	0.2157	1			
7	0.1556	0.1769	0.3887	0.2395	0.3637	0.3677	1		
8	0.2128	0.3322	0.3591	0.3934	0.3607	0.2943	0.3866	1	
9	0.3301	0.2397	0.2145	0.4540	0.4154	0.1661	0.1921	0.3612	1

#### Clean energy

Clean energy refers to energy sources with minimal or negligible adverse environmental effects. Renewable energy sources, including solar, wind, hydro, geothermal, and biomass, are encompassed within this category. Clean energy technologies are meticulously crafted to minimise greenhouse gas emissions, effectively mitigate the adverse effects of climate change, and foster sustainable long-term growth. The transition to clean energy is of utmost importance in reducing dependence on fossil fuels and mitigating the environmental consequences of energy generation and consumption. Table 3 displaced the descriptive statistics, pairwise correlation and VIE.

**Table 3:** Results of descriptive, pair-wise correlation and VIE analyses.

	DF	FD	FDI	GCF	ICT	CE
Mean	7.4793	57.2244	2.935	25.3266	90500000	5.0114
Median	-0.2187	65.0825	1.4034	24.7841	29000000	2.82
Maximum	4.5932	138.8578	32.8243	50.7806	276000000	31.91
Minimum	-4.3467	6.8142	-4.5415	-3.9459	28000000	0
Std. Dev.	1.8266	30.7670	6.0060	9.7481	12367	6.9577
Skewness	0.6678	0.0595	3.4873	0.1392	1.1544	2.0848
Kurtosis	3.5446	2.1167	15.8193	3.9802	2.3331	7.4235
Jarque-Bera	11.5303	4.2032	1393.2435	6.1012	0.9626	229.4246
Observations	320	320	320	320	320	320
Pair-wise correlation						
DF	1					
ICT	-0.0699	1				
ET	0.2313	-0.1202	1			
TO	0.14141	0.0454	0.3730	1		
FO	-0.0525	0.1269	0.0023	0.3328	1	
CE	0.2202	-0.5695	0.2258	-0.0069	-0.2928	1

Output from VIE analysis							
**Scores**	**CE**	**DF**	**ICT**	**FDI**	**ET**	**CGF**	**FD**
**VIF**	1.096	4.9732	1.0466	2.286	4.5254	3.8213	4.4165
**1/VIF**	0.9124	0.201	0.9554	0.4374	0.2209	0.2616	0.2264
**Mean VIF**	3.1664						

### 3.3 Estimation strategy

First is implementing the Cross-sectional dependency test, which is formalized by [87]. Juodis and Reese [87] new cross-sectional dependency [CD], building on Pesaran [88] CD test for residuals from panels with latent factors, which is designed to identify and fix errors caused by cross-sectional dependence in panel data models with latent factors. The latest CSD test demonstrated that it behaves predictably, regardless of whether the latent factors are strong or weak. Even when the latent factors are weak, the test remains reliable and includes a screening component to enhance effectiveness. Their test also tackles the problem of excessive rejection. It can be used with various panel data models, including those with stationary errors and serially correlated errors.

Second, the heterogeneity properties of the research variables were assessed through the execution of the slope of heterogeneity [SHT] introduced by Bersvendsen and Ditzen [89]. Slope of Heterogeneity [SHT] provides numerous advantages over previous methods of measuring the heterogeneity of research data. Compared to prior methodologies, SHT provides a more accurate evaluation of the effect of the examined factors by fully understanding their fluctuations. Furthermore, SHT was created to detect data patterns and variations that traditional approaches might overlook. This considerably enhances the precision and reliability of the analysis. Furthermore, SHT offers a versatile framework for evaluating heterogeneity, making it appropriate for various study settings and data formats. In summary, SHT represents a significant improvement over previous methods for evaluating heterogeneity features, giving researchers a more effective and sophisticated instrument to conduct their investigations.

Third, documenting the variable’s order of integration, the present study has executed the panel unit root test introduced by Herwartz and Siedenburg [90]. Before doing cointegration tests on panel data models with cross-sectional dependency, ensure the variables are stationary. Conventional unit root tests may be invalid when the cross-sectional units are interdependent, as they rely on the assumption that they are independent. Because they are more appropriate for panel data models with cross-sectional dependency and eliminate the necessity for the assumption above, second-generation unit root tests like the Herwartz and Siedenburg [90] tests are often used. The Herwartz and Siedenburg [90] study presupposes the existence of a universal component with uniform effects on every nation. Because of the potential for cross-sectional dependency, this assumption is made. Second-generation tests are preferable when evaluating time series data or tiny cross-sections because they adequately account for any cross-sectional dependency. Evaluations that make it possible to spot patterns of cross-dependence, such as the Pesaran [91] test, can be highly valuable in situations where both cross-sections and time series are limited in size.

Fourthly, over the conventional panel cointegration test, we have executed the novel panel cointegration test proposed by Westerlund and Edgerton [92]. This test is specifically developed to be thorough and adaptable, enabling the detection of cointegration in dependent panels even in the presence of structural failures. The test addresses cross-sectional reliance, which is not considered in first-unit root testing. The Herwartz and Siedenburg [90] test is an example of a second-generation unit root test that is especially suitable for panel data models with cross-sectional dependency. The Westerlund and Edgerton test considers the existence of a shared factor that consistently affects all nations. This factor acknowledges the potential for cross-sectional interdependence. Second-generation tests adequately address possible cross-sectional dependency, making them a more appropriate option for studying tiny cross sections and time series data.

Finally, it explores the magnitudes of independent and control variables: ICT investment, digital financial inclusion, environmental tax, financial openness, trade openness, and environmental quality on clan energy consumption in MEAN nations. The present study has implemented two-panel regression regarding the results derived from CSD and SHT. First, the study implemented Dynamic Common Correlated Effects [DCE] proposed by Chudik and Pesaran [93] and the instrumental variable-adjusted DCE method [DCE-IV from hereafter] recommended by Ditzen [94]. The Dynamic Common Correlated Effects [DCE] model is a highly advanced econometric model widely recognized in time-series analysis. The dynamic correlation effects [DCE] model differs from more traditional approaches since it accounts for the interdependencies and shared correlations across many time series. This method is invaluable to better reflect the dynamics of the actual world’s economy and finances since it captures the changing linkages and interdependence among variables over time. Researchers may improve their predictions and policy suggestions by better comprehending the interrelated nature of economic variables via dynamic, common, correlated effects. DCE has successfully evaluated complex time-series data, yielding important insights for decision-making in many financial and economic contexts.

In addition, Ditzen [94] proposed a major step forward in decision modelling using the instrumental variable-adjusted discrete choice experiment approach [DCE-IV]. Discrete choice experiments [DCEs] are a great way to test hypotheses about endogeneity, but including instrumental variables in DCE-IV makes the findings more accurate and trustworthy. Researchers may more reliably estimate the links under study when they use this method to account for hidden variables that may affect decision-making and the components under study. When evaluating decision-making processes, the DCE-IV framework offers a thorough method that successfully handles biases caused by endogeneity.

## IV. Model estimation and interpretation of the results

Following the framework proposed by Juodis and Reese [87] and Bersvendsen and Ditzen [89], the study assesses the cross-sectional dependency and slope of heterogeneity. Table 4 displays the test statistics with statistical significance. According to test statistics, the study disclosed the presence of CSD and the heterogeneity among the research variables.

**Table 4:** Results of CD and SH test.

Panel A: CD test of Juodis and Reese [2022]							
	**CE**	**DF**	**ICT**	**FDI**	**ET**	**CGF**	**FD**
test stat value	-1.6514	-3.1012	5.5069	5.0031	3.1654	1.9206	4.2221
Probability	**	***	***	***	***	***	***
CD exist	YES	YES	YES	YES	YES	YES	YES
Panel B: SH test of Bersvendsen and Ditzen [2021]							
	Delta	Statistic	Adjusted	Delta	Statistic	SH	exits
Model	3.0199***		5.0292***			Yes	
Model	3.7747***		4.2876***			Yes	

Once CSD and SHT were confirmed, the study implemented Herwartz and Siedenburg [90] in exploring the order of integration and long-run association through Westerlund and Edgerton [92]. The panel unit root test and cointegration results are displayed in Table 5. Referring to the panel unit root test, it is apparent that all the variables become stationary after the first difference, i.e., I [1]. While the cointegration test exposed the rejection of the null hypothesis “no–cointegration”, alternatively unveiling the presence of long-run cointegration between ICT, digital financial inclusion, environmental tax, financial openness, trade openness, and environmental quality in MENA.

**Table 5:** Results from integration and cointegration tests.

Panel A: Integration [or unit-root] test Of Herwartz and Siedenburg Analysis							
	**CE**	**DF**	**ICT**	**ET**	**FO**	**TO**	**EQ**
At a level	0.001	0.3672	-0.1325	0.6019	-0.3145	-0.5491	0.4341
First level	2.9555	-0.0385	0.3026	0.6403	-0.386	1.8004	-2.0289
Panel B: Cointegration test of Westerlund and Edgerton [2008]							
	no shift		mean shift		regime shift		
	LMг	LMΦ	LMг	LMΦ	LMг	LMΦ	
	Stat.	Stat.	Stat.	Stat.	Stat.	Stat.	
Model 1	-4.0978	-4.7245	-2.5262	-4.0749	-3.9937	-3.938	
Model 2	-2.193	-3.8848	-4.1616	-2.3334	-3.2683	-2.7659	

Table 6 displays the results of empirical model execution through DCE and DCE-IV. The coefficients of digital financial inclusion on clean energy have revealed positive and statistical significance in both estimations: DEC [a coefficient of 0.1206] and DCE-IV [a coefficient of 0.1764]. Study findings advocate DF’s contributory effects in the clean energy inclusion process in the energy mix. Our study is in line with existing literature offered by [60, 95, 96]. Using digital inclusive finance may improve the allocation of resources and promote efficient resource consumption, influencing the development of the renewable energy industry [1]. The increased use of digital finance in China has facilitated more investment in the renewable energy industry, exemplifying the characteristics of green finance, enabling the implementation of renewable energy sources via diverse funding options and enhanced energy efficiency [2]. Digital finance alleviates the limitations on funding for renewable energy businesses and individuals, therefore fostering the use of renewable energy in China [3]. By incorporating digital financial technologies like blockchain and mobile payment systems, the availability of green financing options for renewable energy projects is expanded. This leads to enhanced financial inclusion, risk management, and transparency in the renewable energy sector [4, 5].

**Table 6:** Results of empirical model estimation with DCE and DCE-IV.

	Coefficient	Std. Error	t-Stat	Coefficient	Std. Error	t-Statistic
	DCE			DCE-IV		
L. CE[–1]	-0.1383***	0.0305	-4.5344	-0.1327***	0.0232	-5.7219
DF	0.1206***	0.0287	4.2006	0.1764***	0.0425	4.1512
ICT	0.0816**	0.0324	2.5185	0.1405***	0.0355	3.9577
ET	0.2982***	0.0419	7.1186	0.2436***	0.0283	8.6098
FO	0.1072***	0.0189	5.3291	0.1178***	0.0332	3.5506
TO	-0.1463***	0.0296	-4.9429	-0.1614***	0.0295	-5.4732
EQ	-0.0857**	0.0418	2.0514	-0.0964***	0.0167	-5.777
C	-17.089***	0.2401	-71.1656	-13.893***	0.24013	-57.8562

Note: the superscripts of

***, **,* specify the significance level at 1% 5%. And 10% respectively

The coefficients of ICT derived with DCE [a coefficient of 0.0816] and DCE-IV [a coefficient of 0.1405] have been found positive and statistically, indicating Investment in ICT is beneficial for clean energy inclusion in the energy mix. Our study finding is in line with the literature introduced by [45, 46, 97]. ICT investment is crucial for facilitating and encouraging the adoption of renewable energy. Through the utilization of cutting-edge technologies like smart grids, energy storage optimization, predictive analytics, and demand response systems, ICT enables the smooth integration of renewable energy sources into the current energy infrastructure [98, 99]. Technological inclusion facilitates the effective management of renewable energy generation, distribution, and consumption, ultimately resulting in the enhanced utilization of clean and sustainable energy sources [100]. In addition, investing in ICT enables consumers to actively engage in the renewable energy market by utilizing smart devices and energy management systems, which promotes a culture of energy conservation and environmentally conscious consumption [53, 57, 101].

The coefficient of environmental tax in both model estimations, that is, DCE [a coefficient of 0.2982] and DCE-IV [a coefficient of 0.2436], have been found positive and statistically significant at a! level in MENA, suggesting the environmental restriction in terms of the imposition of additional tax act as a catalyst in clean energy inclusion I the energy mix. A similar line of findings can be found in the study of [6, 16, 102, 103]. By promoting the adoption of clean energy and encouraging sustainable practices, environmental taxes can play a crucial role in driving the demand for clean energy and protecting the environment [104]. Clean energy development can significantly contribute to economic growth, particularly in industrialized countries, as long as appropriate environmental charges are put in place [105]. The study of [106], asserted that the Inflation Reduction Act’s tax provisions offer a tax credit for power generation from renewable sources, which can be advantageous for various sectors such as clean energy, automobiles, buildings, and factories. Tax credits for renewable energy are a crucial component of any infrastructure package as they possess the capacity to stimulate substantial climate investments. An effective strategy to mitigate environmental impacts is to employ economic instruments, such as revised taxation policies, to accelerate the shift towards renewable energy sources [107].

Financial openness has exposed a catalyst role in promoting clean energy inclusion in MENA countries; that is, the coefficient of FO established positive and statistically significant in both DCE [a coefficient of 0.1072] and DCE-IV [a coefficient of 0.1178] model estimation. Our study findings are in line with [108, 109]. Foreign direct investment plays a crucial role in facilitating the acquisition of essential capital, technology, and expertise needed to effectively develop and implement clean energy infrastructure [110]. This surge in investment has the potential to expedite the widespread implementation of renewable energy sources like solar, wind, and hydroelectric power. As a result, there will be a significant decrease in our dependence on fossil fuels and a substantial reduction in greenhouse gas emissions. In addition, foreign direct investment [FDI] can play a crucial role in transferring valuable expertise and best practices from established clean energy markets to emerging economies [108, 111]. This exchange of knowledge helps to promote the adoption of sustainable energy consumption on a global level. In addition, implementing financial openness can promote innovation and research within the clean energy industry. This, in turn, can propel the advancement of highly efficient and economically viable renewable energy technologies.

The coefficients of Trade openness [${DCE}_{-0.1463}\;and\;{DCE-IV}_{-0.1614}$] and environmental quality [${DCE}_{-0.0857}\;and\;{DCE-IV}_{-0.0964}$] is negatively linked to clean energy consumption, suggesting that domestic trade liberalization and environmental lethargy in CO2 emission harm clean energy incorporation in the energy mix. Our findings are supported by the literature offered by [112–115]. Research has indicated that the expansion of trade can positively impact GDP and industrial development. However, it is important to note that this growth can also lead to an increase in CO2 emissions resulting from manufacturing processes and energy consumption. The higher emissions are typically attributed to the energy-intensive and reliance on fossil fuels in industrial activities and manufacturing processes associated with commerce. Nevertheless, ample evidence supports the notion of a negative relationship between CO2 emissions and the adoption of renewable energy sources. As a result, we can anticipate a significant reduction in CO2 emissions over time. In addition, the process of trade liberalization can offer countries the opportunity to acquire cleaner energy technology and resources from global markets. This can potentially accelerate the shift towards clean power, which could be particularly beneficial for countries that do not have the resources or necessary infrastructure to produce sustainable energy independently.

Next, the study extended the empirical test considering all nine proxy measures of digital financial inclusion and the results in Table 7. The study documented that proxy measures have mixed effects on clean energy inclusion in MENA countries.

**Table 7:** Robustness estimation with the proxy of digital financial inclusion.

	Coefficient	Std. Error	t-Statistic	Coefficient	Std. Error	t-Statistic
	DCE			DCE-IV		
DF1	0.09849***	0.0322	3.0586	0.07831*	0.0424	1.8469
DF2	-0.0269***	0.0044	-6.0722	-0.0307***	0.00186	16.5053
DF3	-0.0213***	0.0028	-7.4736	-0.0414***	0.00342	-12.1052
DF4	0.0122***	0.0022	5.3275	-0.0096***	0.00261	-3.6781
DF5	0.0367***	0.0017	20.8522	0.0362***	0.00193	18.7564
DF6	0.0242***	0.0032	7.4461	0.042***	0.00275	15.2727
DF7	0.0432***	0.0018	23.2258	0.0019	0.00407	-0.4668
DF8	-0.0422***	0.0021	-19.2694	-0.0119***	0.00239	-4.9790
DF9	0.0353***	0.0033	-10.5688	0.0364***	0.00158	-23.0379
ICT	0.0486***	0.0026	-18.4091	0.0479***	0.00222	-21.5765
ET	0.0117***	0.0017	-6.5730	0.025***	0.00387	-6.4599
FO	0.16138***	0.0191	8.4492	0.14579***	0.046	3.1693
TO	0.08704***	0.0162	5.3728	0.14691***	0.0341	4.3082
EQ	0.10858**	0.0451	2.4075	-0.6920***	0.0281	-24.6270
C	-8.101	0.0309	262.1682	-13.88	0.0214	648.5981

Note: The superscripts of

***, **, and* specify the significance level at 1% and 5%, respectively. And 10% respectively

The following section deals with the country-wise assessment through DOLS and results displayed in Table 8. DF positively affects CE for many of the nations listed, as indicated by the positive coefficients for Algeria, Djibouti, Libya, Morocco, Oman, Qatar, Saudi Arabia, and Tunisia. This is a suggestion digital financial inclusion may result in a favourable ambience in clan energy development of the above-stated MENA nations. ICT also seems to positively affect CE for some nations, such as Algeria, Bahrain, Egypt, Iran, Malta, Morocco, Oman, Qatar, and Saudi Arabia. Study findings postulated that economic progress with ICT growth fosters the speed of renewable energy consumption in the aggregated economy and supports energy efficiency formation. ET shows a positive effect on CE for some nations, including Egypt, Iran, Kuwait, Lebanon, Libya, Malta, Morocco, Oman, and Qatar, suggesting environmental restriction through excessive tax imposition in controlling CO2 emission has assisted in the process of clean energy inclusion in the energy mix. The TO coefficients appear to positively affect CE for some nations, including Algeria, Djibouti, Egypt, Iran, Kuwait, Lebanon, Libya, Malta, Morocco, Oman, Qatar, and Saudi Arabia. Moreover, the finding of FO seems to have a positive effect on CE for some nations, including Algeria, Djibouti, Egypt, Iran, Kuwait, Lebanon, Libya, Malta, Morocco, Oman, Qatar, and Saudi Arabia. Finally, EQ also positively affects CE for some nations, including Algeria, Bahrain, Djibouti, Egypt, Iran, Kuwait, Lebanon, Libya, Malta, Morocco, Oman, Qatar, Saudi Arabia, and Tunisia. Some nations show negative coefficients for certain factors, such as Bahrain for TO, Djibouti for ICT and EQ, Iran for TO, Kuwait for DF, Lebanon for DF, Libya for FO and TO, Qatar for ICT and TO, Saudi Arabia for ICT and TO, Syrian Arab Republic for DF, ICT, and EQ, Tunisia for DF, ICT, and TO, and United Arab Emirates for DF, ICT, and EQ.

**Table 8:** Country-specific assessment: Dynamic OLS.

Nations	DF	ICT	ET	FO	TO	EQ
Algeria	0.155***	0.163***	0.038**	0.067***	0.206**	-0.115***
Bahrain	0.058**	0.257	0.087	-0.011***	0.213***	-0.155***
Djibouti	0.186**	-0.115	0.003	0.147***	0.09**	-0.199***
Egypt, Arab Rep.	0.061***	0.062***	0.145***	0.025***	0.108***	-0.223*
Iran, Islamic Rep.	0.045**	0.227***	0.12***	0.061***	0.064*	-0.137***
Kuwait	-0.024*	-0.069*	0.153**	0.075*	0.218***	-0.251***
Lebanon	-0.005	-0.028	0.014*	0.255*	0.166**	-0.091***
Libya	0.248***	0.072***	0.209***	-0.145***	-0.075*	-0.251***
Malta	0.0410	0.142**	0.107***	-0.018***	0.081***	-0.138*
Morocco	0.202***	0.138***	0.041***	-0.119***	0.201**	-0.166***
Oman	0.186**	0.219*	0.163***	-0.042***	0.169***	-0.175***
Qatar	0.198***	0.0711	-0.012*	0.245**	0.079**	-0.227***
Saudi Arabia	0.151***	-0.112	0.089***	-0.116***	0.188***	-0.246*
Syrian Arab Republic	-0.052***	-0.123	-0.091*	0.059**	0.016***	-0.13***
Tunisia	0.273***	-0.164***	-0.009	-0.077***	0.031*	-0.178***
United Arab Emirates	-0.052***	-0.122***	-0.065	-0.067	0.033*	-0.223***

Note: The superscripts of

***, **, and* specify the significance level at 1% and 5%, respectively. And 10% respectively

## V. Discussion of the study findings

The study findings have revealed that the ICT investment is crucial for facilitating and encouraging the adoption of renewable energy, which is supported by the existing literature [44, 45, 48, 50, 54, 116, 117]. The study of Wang, Qamruzzaman [8], Qamruzzaman and Kler [18], Su, Wang [47], Santarius, Bieser [49] revealed that ICT is crucial in seamlessly incorporating renewable energy sources into the current energy infrastructure; additionally, it empowers consumers by providing them with the necessary information to make well-informed and environmentally conscious energy decisions [45]. ICT facilitates the implementation of advanced smart metering systems, which offer instantaneous information regarding energy usage. Consumers are empowered to closely monitor their energy usage patterns, pinpoint areas for efficiency enhancements, and make well-informed choices regarding integrating renewable energy into their energy consumption habits. ICT solutions enable the integration of energy management systems to maximize the utilization of renewable energy in various settings, including residential, commercial, and industrial environments. These systems can automate energy-saving measures, such as fine-tuning energy consumption following the availability of renewable energy sources. This promotes the increased utilization of clean energy, contributing to a more sustainable future [118, 119].

ICT is critical to integrating renewable energy into Middle Eastern and North African [MENA] energy markets. Individuals, organizations, and communities may efficiently and ethically adopt renewable energy by investing in information and communication technology that provides behavioural insights and feedback mechanisms [54]. Consumers may now actively participate in energy markets, engage in peer-to-peer energy trading, and obtain access to a diversified spectrum of renewable energy sources thanks to the widespread usage of ICT-enabled advanced trading platforms. Energy traders may improve their use of renewable energy sources by exploiting real-time data from modern communication technologies such as Internet of Things [IoT] devices and smart grid systems [56]. Producers may create extra cash by selling surplus energy to clients via energy trading systems. This helps renewable energy providers financially and encourages the broad usage of clean energy sources [55]. Through peer-to-peer energy trading systems, people and corporations may participate in the energy market, which may be accomplished by constructing renewable energy generators, such as solar panels or wind turbines, at their facilities. Nations can create an energy system that is less reliant on centralized utilities and more robust in the face of possible disruptions by distributing power generation [120, 121]. Incorporating ICT into energy trading enables policy implementation monitoring and regular assessment of policy impacts on the use of ICT solutions for energy-efficient management, as well as the development of informative platforms that encourage behavioural changes toward improved energy efficiency.

Investing in information and communication technology may help the Middle East and North Africa [MENA] area promote sustainable energy usage strategies. These devices provide crucial behavioural data and feedback mechanisms that may motivate people to use more sustainable energy. Providing real-time data on energy use and individualized advice may help increase renewable energy adoption. Individuals, for example, may monitor their energy consumption and make educated choices using up-to-date data supplied by smart meters and energy management systems [58]. Furthermore, with the use of mobile apps and web-based platforms, customers may obtain individualized suggestions for lowering energy usage and boosting their use of renewable energy [122], which can also be used to promote ecologically beneficial energy behaviours, such as lowering energy use during peak times or switching to more energy-efficient appliances. Nonetheless, adopting these systems in the MENA region confronts hurdles such as restricted access to ICT infrastructure and low levels of digital literacy. More investment in ICT infrastructure and digital literacy initiatives in the Middle East and North Africa [MENA] is critical [123]. The deployment of ICT in the MENA area has the potential to build a culture of sustainable energy consumption via real-time data on energy use, individualized recommendations, and incentives to encourage sustainable energy consumption practices. Additional investment in ICT infrastructure and digital literacy efforts is required to solve the problems associated with adopting these technologies in the region [117].

The evidence from the empirical assessment suggests that digital financial technologies, such as blockchain, mobile payment systems, and big data analytics, are essential in increasing the accessibility of green funding choices for renewable energy projects. Our study finding is in line with the existing literature offered by [54, 82, 100, 123–125]. Literature postulated that DFI greatly helps the widespread acceptance of renewable energy. Furthermore, the results emphasize the need for continuous governmental backing and budgetary allocations towards digital financial infrastructure to foster a greener and more sustainable energy framework. The study of [126] revealed that China’s shift towards renewable energy sources underscores the substantial impact of green financing and digital finance on the uptake of renewable energy. The significance of digital financial technology in advancing the accessibility of green financing choices for renewable energy projects is emphasized, leading to improved financial inclusion, risk management, and transparency in the renewable energy sector [126]. The study of [65] has advocated for digitally accessible green financing to facilitate the growth of green and renewable energy sources while mitigating CO2 emissions, having the beneficial impact digital money may have on energy resources and endeavours to reduce climate change. [60] suggests that the government could contemplate adopting digital finance rules to get supplementary money for green energy initiatives, which can enhance the use of renewable energy [119].

The study findings support the proposed hypothesis of a positive linkage between digital financial inclusion and clean energy consumption in MENA. Study findings postulate that increasing access to digital financial services may aid the spread of renewable energy across the Middle East and North Africa. This may assist in spreading the word about ecologically friendly and sustainable solutions by simplifying financing for renewable energy projects. Green bonds and carbon credits demonstrate the power of digital finance to direct investments toward environmental sustainability, particularly in renewable energy initiatives [58, 126]. Aside from saving money and accelerating the transfer of funds, digital finance may give more accurate and timely accounting. As a result, renewable energy initiatives may be less expensive than standard energy projects; using the energy business, blockchain technology can boost transaction transparency and tractability [2]. Digital finance can potentially improve access to money for renewable energy projects, especially those on a smaller scale or in a location with few accessible traditional financing sources. Digital finance has the potential to increase involvement in clean energy investment. Crowdfunding and peer-to-peer lending enable a broader spectrum of individuals and organizations to engage in the transition to renewable energy [123]. Digital finance may provide financial support for smart grid technology, energy management systems, and other efficiency-enhancing solutions [122]. Increased access to digital financial services can considerably boost sustainable energy development in the MENA region in the long term; that could be accomplished by increasing the availability of accessible financing options, increasing transparency, and boosting energy efficiency [127].

Digital finance provides effective and transparent financing options for renewable energy initiatives. Investors may easily locate and support renewable energy projects using a range of online platforms and digital technologies, which may lead to a higher cash input into renewable energy projects, hence fostering their development and execution [128]. Digital finance enables the creation of innovative financial tools such as green bonds, carbon credits, and crowdfunding platforms, which provide new avenues to generate funds for clean energy projects and promote the development and use of clean energy technology [129]. Green bonds allow investors to direct their cash towards projects supporting environmental sustainability, such as renewable energy. This serves as an example of how green bonds work [126]. Conversely, carbon credits provide a market-based system to reduce greenhouse gas emissions. Digital finance enhances and streamlines financial transactions, leading to cost savings and faster capital allocation. Clean energy projects may achieve greater economic competitiveness by improving their efficiency compared to traditional energy sources. Furthermore, blockchain technology, a crucial component of digital finance, has the capability to enhance transparency and traceability in energy transactions. It is particularly crucial for renewable energy certificates and carbon trading, since it may provide substantial advantages. Digital finance has the capacity to broaden the availability of cash for clean energy projects, particularly for smaller-scale endeavours and in regions with restricted conventional financing alternatives. Digital finance can enhance accessibility and inclusivity in clean energy investment via crowdfunding platforms and peer-to-peer financing [2, 58, 130].

The study findings of ET effects on clean energy consumption postulated a contributory role that environmental taxes have the potential to play a pivotal role in accelerating the transition to renewable energy sources [131–133]. Governments may successfully encourage companies and people to adopt cleaner and more sustainable energy practices by taxing activities that have negative effects on the environment, such as carbon emissions or the generation of nonrenewable energy, which helps conserve natural resources and promotes the development and widespread use of renewable energy sources [134]. Another factor that has the potential to drastically alter the energy market dynamics is the adoption of environmental levies. Since taxes are driving up the price of traditional energy sources, switching to renewable energy sources is becoming more financially viable [135]. In their respective studies, [136, 137] advocate that ET encourage innovation and draw large investments to the renewable energy industry, opening up new opportunities for business and bolstering the development of existing economies. Incentives and tax credits for producing power from renewable sources, as the Inflation Reduction Act specifies, can dramatically accelerate the adoption of clean energy technology. Additionally, [138] asserted that tax incentives help the environment and promote the development of environmentally friendly transportation, construction, and production methods, which aids in encouraging long-term viability across various economic spheres. Furthermore, renewable energy tax credits may be a powerful tool for encouraging substantial investments in environmentally beneficial projects. Governments have the power to encourage massive public and private investments in renewable energy infrastructure by introducing financial incentives and eliminating cost obstacles, which may help address the effects of climate change while also generating economic benefits, new employment possibilities, and technological breakthroughs. In the study of [139]. An effective plan to move toward a more sustainable and ecologically aware energy system must include the use of economic mechanisms, such as environmental levies and incentives for clean energy. To steer the energy market toward cleaner options, governments should strategically connect economic incentives with environmental goals. This will greatly lessen negative effects on the environment and make a substantial contribution to a greener future [140].

One of the essential strategies to encourage the adoption of renewable energy sources is financial openness, which explains the capacity of a nation to integrate renewable energy sources such as solar, wind, and hydroelectric power into its energy system is determined by its financial accessibility and ability to attract FDI, offering us hope that we may minimize our dependence on fossil fuels and the harm they cause. Foreign direct investment [FDI] in a more established renewable energy industry may also teach developing nations a lot [FDI] [124, 125, 141, 142]. This information sharing contributes to a greater worldwide utilization of renewable energy sources. If enforced, financial transparency may lead to increased investment in renewable energy research and development, leading to more efficient and inexpensive renewable energy systems. Sustainable energy consumption has profited enormously from FDI and other types of financial openness. These elements are critical in aiding the shift to a cleaner, more sustainable energy environment because they give the necessary knowledge and resources. The study’s findings highlight a significant link between trade openness and clean energy consumption, underscoring the influence of international trade practices on environmental considerations in MENA [143–145]. The interplay between these factors raises important questions about the environmental impact of global trade and the potential trade-offs between economic growth and ecological conservation [146]. One possible reason for this negative correlation may be the existence of energy-intensive industries in global trade. Industries frequently prioritize cost efficiency and production scale, occasionally neglecting environmental considerations. Furthermore, the expansion of global trade may lead to unforeseen environmental impacts. For example, the rise in transportation and manufacturing that comes with trade can lead to increased carbon emissions, affecting the use of clean energy. Furthermore, the study’s findings suggest a broader conflict that may arise when striving for economic growth while also considering the imperative of environmental sustainability. Sometimes, the focus on economic development in MEAN through trade can overshadow the significance of prioritizing clean energy consumption and environmental protection [130].

Based on the analysis findings, it can be inferred that carbon emissions hurt the utilization of clean energy. More specifically, as carbon emissions increase, the adoption of clean energy decreases [147]. The inverse relationship between environmental sustainability and carbon emissions underscores the intricate dynamics. Additionally, carbon-intensive behaviours pose significant barriers to the widespread adoption and utilization of cleaner energy sources [148]. Possible factors contributing to this negative impact may include insufficient infrastructure, economic dependence on carbon-intensive industries, and restrictive government regulations in MENA. The potential impact of carbon emissions on clean energy consumption could be worsened by factors such as infrastructure limitations and governmental regulations, which might hinder the widespread adoption of clean energy technologies [149]. Addressing the challenges of climate change and promoting sustainable energy methods requires finding solutions to mitigate this negative impact in MENA. The importance of developing laws and initiatives to reduce carbon emissions and accelerate the shift to renewable energy sources is emphasized. Efforts to reduce carbon emissions from industrial and transportation sectors can involve encouraging the advancement and implementation of clean energy technology, investing in infrastructure for renewable energy sources, and implementing regulatory measures [119, 147].

## VI. Conclusion and policy suggestions

The results of this study offer a comprehensive analysis of the interrelationships among ICT, digital financial technologies, environmental taxes, financial openness, and trade openness and how they impact clean energy consumption in the MENA region.

The key conclusion of the research is that information and communication technology play a critical role in supporting the seamless integration of renewable energy sources into existing energy infrastructure. Customers can regulate their energy use with the aid of ICT since it uses cutting-edge technology and streamlines communication networks. It makes it easier to integrate energy management systems and install sophisticated smart metering systems in various settings, including residential, commercial, and industrial buildings. Furthermore, ICT enables the construction of virtual power plants, consumer interaction platforms, and real-time energy pricing systems. Several breakthroughs are required for renewable energy to attain general acceptance and be utilized in an ecologically responsible way.

Furthermore, it is evident from the research that using digital financial technologies such as blockchain, mobile payment systems, and big data analytics is of utmost importance in expanding the accessibility of green finance options for renewable energy projects. To foster a more environmentally friendly and sustainable energy framework, it is crucial to emphasize the importance of ongoing government support and financial investments in digital financial infrastructure. Green bonds, carbon credits, and crowdfunding platforms exemplify the innovative financial instruments facilitated by digital finance. These instruments play a crucial role in promoting clean energy technology’s expansion and widespread acceptance. Another significant finding from the research is the potential significance of environmental levies in expediting the transition to renewable energy. By aligning economic incentives with environmental objectives, governments have the potential to significantly reduce negative environmental impacts and make substantial contributions to a cleaner future. Environmental levies and clean energy subsidies can raise the expenses associated with traditional energy sources. However, this can also make the shift towards renewable energy more financially viable and attractive. The report emphasizes the significance of financial openness, particularly through foreign direct investment [FDI], in promoting the adoption of renewable energy. Foreign direct investment [FDI] and financial openness are key factors in integrating renewable energy sources, reducing dependence on fossil fuels, and facilitating the exchange of knowledge and best practices between developed and developing clean energy markets.

The study’s findings reveal a notable correlation between trade openness and the utilization of renewable energy, shedding light on the influence of international trading practices on environmental considerations in the MENA region. The importance of striking a balance between economic development and environmental protection is underscored by the need to carefully evaluate the ecological impact of proposed trade laws and practices. Concisely, the study provides a comprehensive analysis that illuminates the various elements influencing the adoption of renewable energy in MENA countries. The findings underscore the importance of implementing strategic policies to tackle the issues arising from carbon emissions and trade-related environmental impacts. It also emphasizes the crucial role of utilizing information and communication technology [ICT], digital financial technology [DFT], environmental taxes, financial openness, and trade openness to encourage the widespread adoption and use of renewable energy sources.

Upon completing a comprehensive examination of the research results, we may provide some policy recommendations for the MENA area to promote renewable energy development. The policy proposals have been meticulously formulated to address the distinct difficulties and possibilities found in the research.

Firstly, Strategic allocation of resources towards Information and Communication Technology [ICT] to facilitate the integration of clean energy, suggesting substantial investment in ICT infrastructure to facilitate the seamless integration of renewable energy sources into the current energy grid. Develop consumer engagement platforms that use information and communication technology [ICT] to educate and inspire consumers to adopt renewable energy usage. These platforms will provide customized energy consumption analysis and incentives for adopting sustainable energy practices.

Secondly, Advocate for the accessibility of eco-friendly finance alternatives for renewable energy initiatives via cutting-edge digital financial technology such as blockchain, mobile payment systems, and big data analytics. Advocate for the significance of government backing and financial provisions for developing digital financial infrastructure, which may significantly enhance the acceptance of renewable energy. Significant insights from successful endeavours in other geographical areas, such as China, may be gleaned. Additionally, promotes the development of innovative financial tools, such as green bonds and crowdfunding platforms via digital finance, helping to attract investments into clean energy projects and facilitate financial inclusion within the sector.

Thirdly, Implement impactful strategies such as environmental levies and tax incentives to accelerate the transition to renewable energy sources. We can incentivize the energy industry to adopt cleaner options by matching the economic incentives with environmental goals. Enacting tax credits and incentives for generating renewable energy while advocating for eco-friendly transportation and building techniques may be successful strategies to encourage substantial investments in clean energy infrastructure.

Fourthly, Promote financial policies that facilitate openness and attract foreign direct investment [FDI] to expedite the incorporation of renewable energy sources such as solar, wind, and hydroelectric power. This will aid in diminishing our dependence on fossil fuels and mitigate greenhouse gas emissions. Utilize the potential of financial transparency to promote the sharing of expertise and information between established clean energy markets and developing economies, fostering innovation and research in the clean energy sector and facilitating sustainable future development.
